# Electroacupuncture in treatment of Parkinson disease: A protocol for meta-analysis and systematic review

**DOI:** 10.1097/MD.0000000000023010

**Published:** 2021-01-22

**Authors:** Cong Gai, Tianyao Qiang, Yuxin Zhang, Yuan Chai, Wandi Feng, Hongmei Sun

**Affiliations:** a Department of Anatomy, School of Preclinical Medicine, Beijing University of Chinese Medicine; b Department of Research and Education, Beijing Ditan Hospital, Capital Medical University; c Department of Integrated Chinese and Western medicine, Northern Sichuan Medical College, Nanchong, Sichuan; d Dongfang Hospital Beijing University of Chinese Medicine, Beijing, China.

**Keywords:** electroacupuncture, meta-analysis, Parkinson disease

## Abstract

**Background:**

Parkinson disease (PD) is a worldwide spread neurodegenerative disorder. Dopamine replacement therapy is currently the mainstream treatment, which can alleviate the symptoms but induces motor complications. Electroacupuncture (EA) is beneficial for PD as an alternative medicine. However, few reliable clinical trials or objective systematic reviews are available to give a verdict on the effectiveness of EA in the treatment of PD. Thus, we evaluate the evidence for EA in PD patients by conducting this meta-analysis.

**Methods:**

PubMed, Cochrane Library, EMBASE, China National Knowledge Infrastructure, Chinese Scientific and Technology Journal database, WanFang Digital Periodicals, and Chinese Biomedical Literature Database (SinoMed) will be systematically searched for evidence by 2 authors individually. The analysis will be conducted by RevMan 5.3 software according to Cochrane Handbook.

**Results:**

The efficacy and safety of EA for PD will be comprehensively assessed from the outcomes, including the effectiveness rate, scores of Unified Parkinson Disease Rating Scale, and Webster scale, superoxide dismutase, lipid peroxides, and dopamine content.

**Conclusion:**

This systematic review will provide evidence for whether EA can treatment PD.

**Registration information:**

PROSPERO CRD42019120956.

## 1 Introduction

Parkinson disease (PD) is the second most common progressive neurodegenerative disorder influencing both motor and nonmotor symptoms.^[1]^ The main pathogenesis of PD is the loss of dopaminergic neurons in the substantia nigra caused by a combination of genetic and environmental factors. At least 6 million people around the world are suffering from PD,^[2]^ and the mean age of diagnosis is 72.4 ± 10 years; men are more vulnerable to develop PD than women.^[3]^ There is no effective treatment to postpone PD progression.^[4]^ Dopaminergic medications are the most effective symptomatic therapy for motor symptoms, in addition, levodopa (L-dopa) is the fundamental choice proved to extend life expectancy. However, long-term L-dopa treatment can lead to motor complications such as the dyskinesias.^[5]^ Thus, there exists a demand for many PD patients seek complementary and alternative therapies for better therapeutic effect.

Acupuncture, a noninvasive procedure, exerts a positive effect in treating patients with PD by stimulating qi and blood to keep balance in the body. When combined with L-dopa, acupuncture improves therapeutic effect, reduced dosage, and alleviates adverse effects of L-dopa.^[6]^ As an indispensable part of acupuncture, electroacupuncture (EA) is a prominent complementary and alternative vehicle for PD patients in relieving motor symptoms, improving nonmotor symptoms such as pain, depression, and autonomic symptoms,^[7]^ and ameliorating activities of daily life.^[8]^ Therapeutic effect of EA may be associated with the following mechanisms. First, EA can alleviate oxidative stress regulating of superoxide dismutase (SOD) and glutathione peroxidase (GSH-Px) activity, GSH contents and malondiadehyde level,^[9]^ reversing the lipid and protein oxidation enhancement.^[10]^ Second, the therapeutic effect of EA is related to the inflammatory response in the pathological process of PD,^[11]^ by down-regulating the expression levels of phosphalized extracellular regulated protein kinases, inflammatory cytokines tumor necrosis factor-α and interleukin-1β proteins,^[12]^ and inflammatory enzyme cyclooxygenase-2.^[13]^ Finally, the action mechanism of EA on treatment may be related with ubiquitin-proteasome system by decreasing alpha-synuclein.^[14]^

However, due to small sample sizes and methodological defects, reliable scientific evidence is absent to prove the therapeutic effect of EA for PD. And among the existing system reviews of acupuncture for PD, manual and electrical acupuncture usually mixed up. In addition, in the preliminary searches of the electronic databases, there was an increase of the studies of EA for PD. Hence, there is a need to conduct the meta-analysis to objectively assess the therapeutic effect, safety, and potential mechanisms of EA in treatment of PD.

## 2 Materials and methods

This study is conducted and reported in accordance with the Preferred Reporting Items for Systematic Reviews and Meta-Analysis Protocol statement guidelines.^[15]^ This review has been registered on PROSPERO international prospective register of systematic reviews (https://www.crd.york.ac.uk/prospero/display_record.php?RecordID=120956), with the registration number: CRD42019120956.

### 2.1 Inclusion and exclusion criteria

#### 2.1.1 Types of studies

Clinical randomized controlled trials (RCTs) taking EA combined with L-dopa therapy for PD will be included.

#### 2.1.2 Types of participants

Patients diagnosed of PD will participant without restrictions of age, gender, race, or duration of disease.

#### 2.1.3 Types of interventions

The intervention of the experiment group will be EA adjuvant with L-dopa, and of the control will be the L-dopa alone.

#### 2.1.4 Types of outcome measures

##### 2.1.4.1 Primary outcomes

(1) Assessment of effectiveness rate;
(2) Overall symptom scores using The Unified Parkinson Disease Rating Scale (UPDRS) and Webster scale;
(3) Motor symptom scores utilizing UPDRS III scale;
(4) Dopamine(DA) content.

##### 2.1.4.2 Secondary outcomes

(1) Nonmotor symptom scores employing UPDRS I scale;
(2) Activities of daily living using UDPRS II;
(3) Complications of treatment applying UPDRS IV;
(4) Antioxidant ability: SOD activity and LPO content;
(5) Content of inflammatory cytokines: tumor necrosis factor-α and interleukin-1β;
(6) Adverse events.

### 2.2 Exclusion criteria

RCTs with any following conditions will be excluded:

(1) Duplicated publications;
(2) Participants diagnosed with a parkinsonian syndrome or with severe complications;
(3) Combined with other therapy.

### 2.3 Search strategy

Electronic literature search will be performed using PubMed, the Cochrane Library, Embase, China National Knowledge Infrastructure, Chinese Scientific and Technology Journal database, WanFang Database, and Chinese BioMedical Literature Database (SinoMed) for English and Chinese articles by March 24, 2020. Search terms will be used individually or in combination. English search terms comprise Parkinson's disease, Parkinson disease, Parkinsons disease, Parkinsonism, acupuncture, acupuncture therapy, acupuncture points, electroacupuncture, electrical acupuncture, electro-acupuncture, electro acupuncture, randomly, randomized, and clinical trial, Chinese search terms included generic names for PD (Pa jin sen or Zhen chan ma bi), EA (Dian zhen), randomized (Sui ji) and control (Dui zhao). Additional searches in the light of relevant systematic reviews will also be manually performed to make the search comprehensive. In addition, WHO International Clinical Trials Registry Platform, ClinicalTrials.gov, and the Chinese Clinical Trial Registry will be searched. For ongoing trials, author will be contacted for relevant data. The search strategy for PubMed is shown in Table 1.

**Table 1:** Search strategy.

Number	Search terms
1	Exp acupuncture or acupuncture therapy or Acupuncture Points or electroacupuncture
2	Acupuncture. ti, ab.
3	Acupuncture therapy. ti, ab.
4	Acupuncture Points. ti, ab.
5	Electroacupuncture. ti, ab.
6	Electric acupuncture. ti, ab.
7	Electrical acupuncture. ti, ab.
8	Electro-acupuncture. ti, ab.
9	Electro acupuncture. ti, ab.
10	Or 1–9
11	Exp parkinson disease. ti, ab.
12	Parkinson's disease. ti, ab.
13	Parkinson disease. ti, ab.
14	Parkinsons disease. ti, ab.
15	Or 11–14
16	Controlled clinical trial. pt.
17	Randomized controlled trial. pt.
18	Randomized. ab.
19	Randomly. ab.
20	Trial. ab.
21	Or 16–20
22	Exp animals/not humans. sh.
23	21 not 22
24	10 and 15 and 23

### 2.4 Data collection and analysis

#### 2.4.1 Selection of studies

All authors will be trained to reduce human factors in carrying out this review. During search period, EndNote X8.2 will be used for records management. According to the predetermined inclusion and exclusion criteria, 2 authors (Tianyao Qiang and Yuxin Zhang) will screened studies separately by title, keywords, abstracts, and full texts if needed. Each article excluded will be given a reason and recorded in summary. Any discrepancy will be resolved through discussion or consultation a third author (Cong Gai). The selection process will be detailed in the Preferred Reporting Items for Systematic Reviews and Meta-Analysis flow chart shown in Figure 1.

**Figure 1:** Flow diagram of the study selection process.

#### 2.4.2 Data extraction and management

Two authors (Tianyao Qiang and Yuan Chai) will separately extract the important data, according to a premade collection form. If discrepancies encountered, a consensus will be reached by consulting an expert reviewer (Cong Gai). If the data needed in the records were not given, we will contact the author for more. The following information will be extracted: study details (authors, country, publication time, journal name, title, contact information), participants (inclusion and exclusion criteria, PD diagnostic criteria, age, gender, race, disease duration, baseline data), study methods (registry platform, sample size, blinding method, randomization method, allocation concealment, incomplete report or selecting report), the interventions (type of acupuncture, needles, acupoints, electric frequency, treatment duration, treatment frequency, practitioner, dosage of L-dopa) and the outcomes (primary and secondary outcomes shown above).

#### 2.4.3 Risk of bias assessment

The following 7 domains of Cochrane Handbook for Systematic Reviews will be applied to assess the risk of bias by 2 authors (Yuxin Zhang and Yuan Chai) independently: randomized sequence generation, allocation concealment, blinding of participants, personnel and outcome assessors, incomplete outcome data addressed, selective reporting, and other issue. On this account, the incorporated literature will be divided into 3 categories: low risk, high risk, and unclear. In the event of a divergence, discussion will be conducted. If no agreement can be reached a third party (Wandi Feng) is consulted for consensus.

#### 2.4.4 Data synthesis

Data analysis will be carried out using RevMan 5.3 software. Dichotomous data will be presented as relative risks, continuous variables measuring with the same scale will be presented as with mean differences or the standardized mean differences. Effect sizes will be indicated by 95% confidence intervals.

#### 2.4.5 Unit of analysis issues

If multiple interventions are included, we will combine EA groups as the experimental group; if multiple groups using L-dopa plus EA, we will combined them into 1 group as control.

#### 2.4.6 Dealing with missing data

If the data information of the included trials are found to be incomplete, 2 authors (Tianyao Qiang and Wandi Feng) will contact the first authors and the corresponding authors by email. The unobtainable data will be excluded and only the complete data will be analyzed. In addition, the reason for the missing of the data and the impact for the analysis will be discussed.

#### 2.4.7 Assessment of heterogeneity

Heterogeneity among studies is tested via chi-square test and *I*^2^ statistic tests. *P* < .05 and *I*^2^ > 50% indicated the existence of heterogeneity. Fixed-effect models are applied if there was no significant heterogeneity across studies (*I*^2^ < 50%); otherwise, random-effects models were applied.

#### 2.4.8 Assessment of publication bias

If more than 10 articles are included, the funnel plot of Revman 5.3 software is used to analyze publication bias. The symmetrical distribution on both sides of funnel plot data indicates that there is no publication bias, while the asymmetry on both sides may lead to publication bias. If the number of articles is less than 10, the Egger test and Begg test of Stata 14.0 software are used for statistical analysis. *P* < .05 indicates the existence of publication bias, while *P* > .05 indicates the absence of publication bias.

#### 2.4.9 Subgroup analysis

Subgroup analysis is conducted based on intervention time, gender, age and quality score of included literature, and efficiency is taken as the basis.

#### 2.4.10 Sensitivity analysis

Sensitivity analysis is performed when there are important positive results or critical results in primary analysis. After excluding abnormal results (too large or too small samples), meta-analysis was conducted to consider whether there was any change. If there is no significant difference between the results before and after sensitivity analysis, the results are proved to be stable.

#### 2.4.11 Grading the quality of evidence

According to the GRADE, the evidence quality is divided into 4 grades: high, medium, low, and extremely low.

### 2.5 Data analysis

Subgroup analysis by intervention duration is conducted in effectiveness rate. Publication bias is assessed by funnel plots for more clinically instructive.

### 2.6 Ethics and dissemination

The ethics approval is not needed as the data are extracted from the published literature and they are not related to the individual patient's data. This systematic review and meta-analysis will be published in a peer-reviewed journal

## 3 Discussion

PD is a common neurodegenerative disease, the main clinical manifestations are static tremor, muscle stiffness, bradykinesia, and postural balance disorders. EA is considered as a non-drug treatment method for PD,^[16,17]^ with the advantages of simple operation, convenience, and fewer side effects. At present, it is not clear whether EA combined with L-dopa is better than L-dopa alone in the treatment of PD. This study will conduct a meta-analysis of the relevant RCT, and comprehensively evaluate the efficacy and safety of EA in the treatment of PD through the effective rate, UPDRS score, Webster score, SOD, LPO and DA contents, so as to provide evidence for the treatment of PD and better guide clinical practice.

## Author contributions

**Conceptualization:** Cong Gai, Hongmei Sun.

**Data curation:** Tianyao Qiang, Yuxin Zhang, Yuan Chai.

**Formal analysis:** Tianyao Qiang, Yuxin Zhang, Yuan Chai.

**Funding acquisition:** Cong Gai, Hongmei Sun.

**Investigation:** Tianyao Qiang, Yuxin Zhang, Yuan Chai.

**Methodology:** Cong Gai, Hongmei Sun.

**Project administration:** Tianyao Qiang, Yuxin Zhang, Hongmei Sun.

**Resources:** Cong Gai, Tianyao Qiang, Hongmei Sun.

**Software:** Tianyao Qiang, Yuxin Zhang, Wandi Feng.

**Supervision:** Tianyao Qiang, Yuxin Zhang, Yuan Chai, Wandi Feng, Hongmei Sun.

**Validation:** Cong Gai, Tianyao Qiang, Yuxin Zhang, Wandi Feng, Hongmei Sun.

**Visualization:** Tianyao Qiang, Wandi Feng.

**Writing – original draft:** Cong Gai, Tianyao Qiang, Yuxin Zhang, Yuan Chai, Wandi Feng, Hongmei Sun.

**Writing – review & editing:** Cong Gai, Tianyao Qiang, Yuxin Zhang, Yuan Chai, Wandi Feng, Hongmei Sun.
